The article "Spectral-Spatial Attention Transformer with Dense Connection for Hyperspectral Image Classification" was published in 2022. Journal: Comput Intell Neurosci.

# Spectral-Spatial Attention Transformer with Dense Connection for Hyperspectral Image Classification

**DOI:** 10.1155/2022/7071485

**Published:** 2022-05-26

**Authors:** Lanxue Dang, Libo Weng, Weichuan Dong, Shenshen Li, Yane Hou

**Affiliations:** ^1^School of Computer and Information Engineering, Henan University, Kaifeng, China; ^2^Department of Geography, Kent State University, Kent, OH, USA; ^3^Aerospace Information Research Institute, Chinese Academy of Sciences, Beijing, China

## Abstract

In recent years, deep learning has been widely used in hyperspectral image (HSI) classification and has shown good capabilities. Particularly, the use of convolutional neural network (CNN) in HSI classification has achieved attractive performance. However, HSI contains a lot of redundant information, and the CNN-based model is limited by the receptive field of CNN and cannot balance the performance and depth of the model. Furthermore, considering that HSI can be regarded as sequence data, CNN-based models cannot mine sequence features well. In this paper, we propose a model named SSA-Transformer to address the above problems and extract spectral-spatial features of HSI more efficiently. The SSA-Transformer model combines a modified CNN-based spectral-spatial attention mechanism and a self-attention-based transformer with dense connection. The SSA-Transformer model can combine the local and global features of HSI to improve the performance of the model. A series of experiments showed that the SSA-Transformer achieved competitive classification accuracy compared with other CNN-based classification methods using three HSI datasets: University of Pavia (PU), Salinas (SA), and Kennedy Space Center (KSC).

## 1. Introduction

Hyperspectral image (HSI) contains rich information in both spectral and spatial dimensions with high correlation [1, 2]. Based on such advantages, HSI has been applied in many fields, such as mineral exploration, environmental monitoring, and urban development. So far, much effort has been made in the field of HSI analysis and processing, including classification [3], anomaly detection [4, 5], and dimensionality reduction [6]. Previous studies of HSI classification mostly used support vector machines (SVM) [7–9], k-nearest neighbor (k-NN) [10], and multinomial logistic regression (MLR) [11]. However, these models heavily rely on experts' domain knowledge and engineering experience.

With the development of deep learning methodologies, multiple HSI classification methods have been developed and widely used in the past few years, including Stacked Autoencoder (SAE) [12], Deep Belief Network (DBN) [13–15], and Recurrent Neural Network (RNN) [16, 17]. In addition, CNN has the advantages of directly processing 3D image patches and extracting a large amount of spatial context information, so a large number of CNN-based models have appeared in the field of HSI classification [18–23]. Hu et al. [18] used convolutional neural networks for HSI classification for the first time. However, the model only contains 1D convolution kernels, so only spectral information of HSI is used in classification and does not consider the spatial context information of HSI, which could potentially impact the accuracy of the model. Later, various models have emerged that use both spatial and spectral information for classification. He et al. [19] used multiple 3D convolution kernels of different sizes to build an M3D-DCNN model, which can extract multiscale spectral-spatial information on HSI. Gao et al. [20] used the small convolution and dense connection in their model to extract spectral-spatial features. The depth of the above model is shallow, and the performance of the model is not good enough. The CNN-based model can extract more rich features by deepening the depth of the model. Paoletti et al. [21] proposed a deep residual network (pResNet) by stacking the pyramid bottleneck residual units derived from the pyramid residual network [24]. The depth of the model can reach more than 30 layers, which can extract rich spectral feature and spatial feature. This model contains a large number of 2D convolution kernels, and the performance of the model is much better than the above models, but as the depth of the model becomes deeper, the training time becomes longer. Li et al. [22] proposed a dual-branch network to extract spectral and spatial information separately; however, stacking multiple 3D convolution kernels also caused the model training time to be too long, and the performance of the model did not improve much. The receptive field of CNN is limited by the small-sized convolution kernel. As a result, the CNN-based model cannot extract global features, which causes a bottleneck in the performance of the CNN-based model.

The article "Spectral-Spatial Attention Transformer with Dense Connection for Hyperspectral Image Classification" was published in 2022. Journal: Comput Intell Neurosci.

To solve the above problems, many transformer-based models have emerged. Considering the large spectral dimension of HSI, HSI can be regarded as sequence data. Just as the word vector in the NLP field represents the meaning of a word, the spectral vector of the HSI pixel represents land cover information. Moreover, the spatial information of HSI is similar to the context of the target word in the NLP field [25]. The transformer model was originally used in natural language processing (NLP) [26–28]; the self-attention mechanism of this model can mine the global features of the sequence, which makes it a great success in the field of NLP. The use of self-attention-based transformer model can make better use of the correlation of HSI information and can extract the global features of neighborhood pixel blocks. However, the performance of many transformer-based models is still not good enough. The model proposed by Hu et al. [29] combines 1D-CNN and Vision Transformer (ViT) [30], but the overall accuracy on PU and SA datasets is only 93.77% and 96.15%, respectively. The reason is that ViT directly segments the input image and cannot handle the low-level features of the input image well [31]. Inspired by the model proposed by Yuan et al. [31], we use a spectral-spatial attention mechanism to process neighborhood pixel blocks to obtain feature maps and then segment the feature maps. In this study, we propose a model that combines a CNN-based spectral-spatial attention mechanism and a self-attention-based transformer (SSA-Transformer). The advantage of the SSA-Transformer is that it can extract local and global features of HSI data and improve classification results. Specifically, the spectral-spatial attention mechanism is used to extract the local features of the neighborhood pixel blocks, reduce redundant information, then process them into sequences, and finally extract the global features by the self-attention-based transformer encoder block. We compared the proposed SSA-Transformer with other CNN-based methods on three HSI public datasets revealing its competitive classification performance.

The main contributions of this work can be summarized as follows:

1. In our proposed model, we use a spectral-spatial attention mechanism to extract the low-level features of the neighborhood pixel blocks, which solves the disadvantage that the transformer part of the model cannot extract the rich low-level features of the input image.
2. Our model combines the advantages of both CNN and transformer. The local features of HSI can be extracted through the CNN part of the model, while the global features of HSI can be extracted through the transformer part of the model. Therefore, the model can effectively extract the local and global features of HSI for more efficient classification.
3. We applied dense connection to connect the extracted features of each transformer encoder block directly to all subsequent transformer encoder blocks to further improve the flow of information among transformer encoder blocks and reduce information loss.

## 2. Methodology

In this section, we first explain the details of the spectral-spatial attention mechanism. Next, we introduce the principles of linear embedding and transformer encoder. Finally, we discuss the overall architecture of the proposed HSI classification method.

The article "Spectral-Spatial Attention Transformer with Dense Connection for Hyperspectral Image Classification" was published in 2022. Journal: Comput Intell Neurosci.

### 2.1. Spectral-Spatial Attention

The transformer-only model will directly segment the input image, but this will cause the model to fail to extract rich low-level features. Therefore, we use the attention mechanism to extract the rich low-level features of the neighborhood pixel blocks of the input model. Specifically, we use the modified CBAM [32] as the spectral-spatial attention mechanism for feature extraction of neighborhood pixel blocks. The spectral-spatial attention module consists of a spectral attention module (SeAM) and a spatial attention module (SaAM) [33]. SeAM is used to select spectral features that are useful for classification, while SaAM is used to select spatial features that are useful for classification.

Figure 1 shows the structure of the entire spectral-spatial attention mechanism. We first utilize convolution operations on the HSI neighborhood pixel block *y* ∈ *R*^*H*×*H*×*C*^, where *H* and *C* represent the spatial size and the spectral dimension, respectively. Next, we extract features in the input data that contribute to classification by SeAM and SaAM, respectively. Note that none of these steps change *C*. Finally, 1 × 1 Conv is used to extract discriminative features on the neighborhood pixel blocks and reduce the number of dimensions of the spectral dimension. During this process, useless information is discarded to avoid the risks of reducing classification performance. We will introduce the detailed process of the spectral-spatial attention mechanism in the next section. The overall attention calculation can be summarized as follows:

(1) $$\begin{array}{c} y^{\prime }=\text{Conv}1\left(y\right),\\ y^{\prime \prime }=M_{se}\left(y^{\prime }\right)*y^{\prime },\\ y^{\prime \prime \prime }=M_{sa}\left(y^{\prime \prime }\right)*y^{\prime \prime }+y,\\ y^{\prime \prime \prime \prime }=\text{Conv}2\left(y^{\prime \prime \prime }\right), \end{array}$$

where *∗* denotes the elementwise multiplication, Conv1() consists of two 3 × 3 convolution layer, *M*_*se*_( ) denotes the spectral attention module, *M*_*sa*_( ) denotes the spatial attention module, and Conv2( ) consists of one 1 × 1 convolution layer.

### 2.2. Spectral Attention Module

For different classes of pixels in HSI, the spectral bands that contribute to the classification are different, and some spectral bands will reduce the accuracy of the classification [34]. Therefore, the role of SeAM is to strengthen the contribution of the spectral bands that are helpful to the classification and weaken the contribution of the spectral bands that are useless or even harmful to the classification. This module maps the input into a weight vector to indicate the contribution of each spectral band to the classification result.

The article "Spectral-Spatial Attention Transformer with Dense Connection for Hyperspectral Image Classification" was published in 2022. Journal: Comput Intell Neurosci.

The structure of SeAM is shown in Figure 2. The module first generates two 1 × 1 × C vectors, *P*_*s*e_^avg^ and *P*_*s*e_^max^, *P*_*s*e_^*avg*^ is generated by global average pooling, and *P*_*s*e_^max^ is generated by global max pooling. After that, the two vectors are first passed through the *F*1 fully connected layer for dimensionality reduction, and then the dimensionality is restored through the *F*2 fully connected layer. Next, the spectral weight vector *P*_*se*_ is generated by the addition of these two vectors and processed by the ReLU activation function. *P*_*s*e_ is calculated by

(2) $$\begin{array}{c} P_{se}{}^{\prime }=F_{2}\left(\sigma \left(F_{1}\left(P_{se}^{\text{avg}}\right)\right)\right)+F_{2}\left(\sigma \left(F_{1}\left(P_{se}^{\max}\right)\right)\right),\\ P_{s\text{e}}=\text{sigmoid}\left(P_{s\text{e}}{}^{\prime }\right), \end{array}$$

where *σ* denotes the ReLU activation function.

Finally, the spectral weight vector *P*_*se*_ is multiplied by the input spectralwise to get the output *y*^″^.

(3) $$\begin{array}{c} y^{\prime \prime }=P_{s\text{e}}*y^{\prime }. \end{array}$$

### 2.3. Spatial Attention Module

All pixels of a neighborhood block are initially considered to be the class of the center pixel; that is, the contribution of all neighbor pixels to the class of the center pixel is initially the same [33]. However, there is no way to distinguish the contributions of different pixels in the neighborhood, which may affect the classification of pixels located on the boundary between two different categories. In addition, not all pixels in the neighborhood contribute to the classification of the center pixel, and some of them may even reduce the classification effect [33]. Therefore, the role of SaAM is to enhance the contribution of pixels that are helpful for classification and weaken the contribution of pixels that are useless or even interfere with the classification. The structure of SaAM is shown in Figure 3. This module first calculates the average value and maximum value of the elements of the spectral dimension, respectively, and obtains the outputs *P*_*sa*_^avg^ and *P*_*sa*_^max^ with the shape of *H* × *M* × 1.

Next, we concatenate these two outputs and go through a convolution operation and a sigmoid activation function to get a new output, which represents the contribution of each pixel. The specific calculation process is as follows:

(4) $$\begin{array}{c} P_{s\text{e}}{}^{\prime }=\text{conv}\left(\left[P_{sa}^{\text{avg}},P_{sa}^{\text{max}}\right]\right),\\ P_{s\text{e}}=\text{sigmoid}\left(P_{s\text{e}}{}^{\prime }\right). \end{array}$$

Finally, *P*_*s*e_ is multiplied by the input spatialwise to get the output *y*^′″^.

(5) $$\begin{array}{c} y^{\prime \prime \prime }=P_{sa}*y^{\prime \prime }. \end{array}$$

The article "Spectral-Spatial Attention Transformer with Dense Connection for Hyperspectral Image Classification" was published in 2022. Journal: Comput Intell Neurosci.

### 2.4. Linear Embedding

Transformer abandons the sequence dependency characteristics of RNNs and introduces a self-attention mechanism. The self-attention mechanism can capture the global information (long-term correlation) of the input patch at any location [35]. But it will cause the input vector to lose the positional relationship. Therefore, ViT solves this problem by processing the sequence into a linear embedding sequence [30]. The overall process is shown in Figure 4: first segment the input data into patches, then flatten it into vectors, then add an extra vector for classification, and finally add a position code to each vector.

### 2.5. Transformer Encoder Block

Inspired by transformer [36], Vision Transformer [30] based on self-attention has successfully applied it in the field of computer vision. The self-attention mechanism in the transformer model can extract global features, which is the key to its attractive effect [30].

Figure 5 shows the architecture of the transformer encoder block, each of which consists of a multihead self-attention mechanism sublayer and a feedforward network sublayer. Residual connections are used between each sublayer and normalize the input of each sublayer using LayerNorm (LN). Self-attention mechanism can be defined as

(6) $$\begin{array}{c} \text{Attention}\left(Q,K,V\right)=\text{soft}\max\left(\frac{Qk^{T}}{\sqrt{d_{k}}}\right)V, \end{array}$$

where *k*, *Q*, *V*, and the output are matrices. *K*, *Q*, and *V* are obtained by multiplying the input matrix by *w*^*Q*^, *w*^*K*^, and  *w*^*V*^ matrices. Use the dimension d_*k*_ of *Q* to participate in scaling.

Note that this is not the only self-attention mechanism in each transformer encoder block. There are multiple such self-attention mechanisms, which constitute a multihead self-attention mechanism. Finally, we define the multihead self-attention mechanism as

(7) $$\begin{array}{c} \text{Multi}-\text{Head attention}\left(Q,K,V\right)=\text{concat}\left({\text{Attention}}_{1},{\text{Attention}}_{2}\text{,…},{\text{Attention}}_{h}\right)W^{o}, \end{array}$$

where *W*^*o*^ is a weight matrix and *h* is the number of the heads.

The feedforward network in each transformer encoder block consists of two full connection layers and a GeLU activation function, which can be defined as

(8) $$\begin{array}{c} \text{FFC}\left(\text{input}\right)=\text{FC}.\left(\sigma \left(\text{FC}\left(\text{input}\right)\right)\right), \end{array}$$

where *σ* denotes the GeLU activation function.

The article "Spectral-Spatial Attention Transformer with Dense Connection for Hyperspectral Image Classification" was published in 2022. Journal: Comput Intell Neurosci.

### 2.6. Overview of the Proposed Model

Figure 6 shows the overall architecture of our proposed model. First, we take each labeled pixel as the center to extract a neighborhood pixel block of size *h* × *h* × *c*, where *h* is the length and width of the pixel block and *c* is the spectral dimension of different HSIs. We use padding operations for edge pixels that cannot be directly extracted into pixel blocks. Finally, we get sample data of shape (*n*, *h*, *h*, *c*), where *n* is the total number of samples.

Then, we use the spectral-spatial attention module to extract the spatial and spectral features of the sample data and reduce redundant information. The spectral-spatial attention mechanism reduces the redundant information of the input data in the spectral band, and the shape of the output data is (*n*, *h*, *h*, *k*), where *k* is the number of spectral bands retained by the data after processing through a 1 × 1 convolutional layer.

Next, we segment each output data with shape (*h*, *h*, *k*) into (*h* × *h*)/(*p* × *p*) patches with shape (*p*, *p*, *k*). We set *p* to 3. The patches of shape (*p*, *p*, *k*) will be reshaped into a one-dimensional vector of length *k* × *P* × *P*. The shape of the data can be redefined as (*N*, *D*), where *N* is the length of the sequence, the size is (*h* × *h*)/(*p* × *p*), *D* is the dimension of each vector of the sequence, and the size is *p* × *p* × *k*.

Finally, by adding the embedding vector and the position code, we finally create a matrix of size (batch size, *N* + 1, *D*) to use as the input to the transformer part of our model. We use multiple transformer encoder modules to continuously extract image features and use the dense connection structure to reduce the loss of information.

## 3. Experiments

In this section, we first introduce these three HSI datasets used to measure the performance of the model: Kennedy Space Center (KSC), University of Pavia (PU), and Salinas (SA), as illustrated in Figures 7–9. The details of the datasets are shown in Table 1. Next, we specify the model configuration process. Finally, we analyze the four factors that affect the performance of the proposed model. We choose overall accuracy (OA), average accuracy (AA), and KAPPA coefficient (*κ*) as the measurement indices of SSA-Transformer performance.

In Salinas dataset, we randomly selected 10% of the dataset for training for our experiments. In Kennedy Space Center dataset, we randomly selected 200 samples per class object as the training set. In University of Pavia dataset, we randomly selected 400 samples per class object as the training set. A detailed experimental analysis is presented in this section. When the number of labels in some categories of the dataset is too small to be selected, 80% of the total number of labels in this category are selected as the training set. We randomly take out 25% of the training set to serve as the validation set. To be fair, we used randomly selected training data for ten experiments in all subsequent experiments and presented the mean and standard deviation of the experimental results.

The article "Spectral-Spatial Attention Transformer with Dense Connection for Hyperspectral Image Classification" was published in 2022. Journal: Comput Intell Neurosci.

### 3.1. Experimental Datasets

*Kennedy Space Center (KSC)*. This dataset was collected by Airborne Visible/Infrared Imaging Spectrometer (AVIRIS) sensors in the Kennedy Space Center. It has a total of 224 spectral bands. After removing the water absorption and low signal-to-noise ratio (SNR) bands, the remaining 176 bands are used for experiments. Its size is 512 × 614 pixels, with a total of 5,211 marked pixels and 13 land cover categories.  Table 2 lists the specific division of the dataset.

*University of Pavia (PU)*. This dataset was collected by ROSIS sensors in the urban area of the University of Pavia in northern Italy. It has 115 spectral bands. After removing the bands affected by noise, 103 bands are left for experiments. It has a size of 610 × 340 pixels, a total of 42,776 marked pixels, and 9 land cover categories.  Table 3 lists the specific division of the dataset.

*Salinas (SA)*. This dataset is acquired by the AVIRIS sensor. The database has 224 spectral bands, with 20 water absorption bands removed, leaving 204 bands for experiments. The size of Salinas is 512 × 217 pixels. There are a total of 54,128 marked pixels and 16 land cover categories.  Table 4 lists the specific division of the dataset.

### 3.2. Experimental Configuration

To evaluate the performance of the model proposed in this paper, the experiments are implemented on a computer with an AMD CPU R7-4800 at 2.9 GHz, a memory size of 16 GB, and an RTX2060 graphical processing unit (GPU).

The model proposed in this paper was implemented by Python version 3.7.0 and the deep learning framework of PyTorch version 1.2.0. Optimization is performed by SGD optimizer [37]. The loss function of our proposed model uses the cross-entropy function. In the experiment on the PU dataset, the learning rate is set to 0.01, and it decays to 0.001 in the 41st epoch. In the experiment on the SA dataset, the learning rate is set to 0.005, which decays to 0.001 at the 41st epoch and decays to 0.0001 at the 81st epoch. In the experiment on the KSC dataset, the learning rate is set to 0.01, decays to 0.001 at the 41st epoch, and decays to 0.0001 at the 81st epoch.

### 3.3. Parameter Setting

Some factors have a significant impact on the classification performance of the model, and we analyze the impact of these factors on the model in this subsection. These factors are batch size, spatial size, training sample, and the number of heads of multihead self-attention. The total epochs of the three dataset experiments of PU, SA, and KSC are set to 80, 120, and 120, respectively.

The article "Spectral-Spatial Attention Transformer with Dense Connection for Hyperspectral Image Classification" was published in 2022. Journal: Comput Intell Neurosci.

#### 3.3.1. Batch Size

A batch size matching the model can effectively improve the accuracy of the model and improve memory utilization. We test the accuracy of the model when the batch size is 16, 32, and 64 with results shown in Figure 10. Our experiments show that when the batch size of the SA, PU, and KSC datasets is all 64, the model performs the best for classification on the three datasets.

#### 3.3.2. Spatial Sizes

The spatial sizes determine the spatial information that the model can use for classification and has a great impact on the performance of the model. To evaluate the impact of the spatial size on the performance of the SSA-Transformer, we choose the spatial size of 9, 15, and 21 for the experiment.  Figure 11 shows the performance (OA) of the spatial size on the SSA-Transformer. We observed that as the spatial size increases, the accuracy of the model did not necessarily increase. This is because as the spatial information increase, there will be more pixels interfering with the classification.

Considering that larger spatial sizes will lead to higher computational costs, the spatial sizes of SA, PU, and KSC datasets are set to 9×9, 15×15, and 9×9, respectively.

#### 3.3.3. Training Sample

We consider utilizing 5%, 10%, and 15% of the sample data in SA and 200, 300, and 400 samples per class in KSC and PU as the training set, respectively. The rest of the data is used as the test set. Figure 5 shows the results obtained by training our proposed model on the corresponding sample dataset. From Table 5, we can see that, in the experiment on KSC, the accuracy of the three sets of data is not much different. The experiments on the remaining two datasets are that the larger the training set, the higher the accuracy. The reason is that the training set can alleviate the overfitting problem of the model.

There is a trade-off between the performance and training time of the model. For the Pavia University dataset, we employ a 400 per class strategy. For KSC, we employ a 200 per class strategy. For Salinas, we employ 10% of the sample data.

#### 3.3.4. The Number of Heads of the Multihead Self-Attention Mechanism

The multihead self-attention mechanism can focus on different positions and can more effectively mine the relationship between the various vectors of the sequence. Therefore, we choose head = 4, 6, and 8 for the experiment.  Figure 12 shows the effect of different number of heads on the accuracy of the model. There is a trade-off between the performance and training time of the model. The number of heads of SA, PU, and KSC datasets is set to 8, 6, and 8, respectively.

The article "Spectral-Spatial Attention Transformer with Dense Connection for Hyperspectral Image Classification" was published in 2022. Journal: Comput Intell Neurosci.

## 4. Results and Discussion

In this section, we used several recently developed typical CNN-based models to measure the performance of our proposed model, including 1D-CNN [18], M3D-DCNN [19], SC-FR [20], pResNet [21], and DBDA [22]. We repeat all experiments in the three datasets 10 times to ensure the fairness of the experiment. We uniformly use the spatial size, training sample, and batch size determined in Section 3 as the input of the comparison model and the model we proposed. The evaluation indicators OA, AA, and KAPPA coefficients are expressed in the form of “mean ± standard deviation.” In addition, we also use the variance of OA and the variance of AA to express the volatility of accuracy.

### 4.1. Comparing with Other Methods

The classification results for each of the methods are shown in Tables 6–8. Experimental results demonstrate that our proposed model achieves the best performance on the PU and SA datasets. On the KSC dataset, compared with DBDA, our proposed model is 0.01%, 0.01%, and 0.02% lower than OA, AA, and KAPPA, respectively, but the gap is not significant. For the proposed model, in the Salinas dataset, compared with 1D-CNN, the OA, AA, and KAPPA of our model are 10.02%, 9.36%, and 13.42% higher, respectively. This is because 1D-CNN does not only extract the spatial feature of HSI but only extract the spectral feature of HSI. M3D-DCNN, pResNet, and SC-FR are models based on 3D pixel blocks that do not use the attention mechanism. M3D-DCNN uses a variety of convolution kernels of different sizes to obtain multiscale information. Even if 3D convolution is used, since the attention mechanism is not used, the OA, AA, and KAPPA are 3%, 1.55%, and 3.34% lower on the Salinas dataset compared with our proposed model, respectively. pResNet and SC-FR are 2DCNN-based models, but compared to our proposed model, OA is 0.04% and 1.18% lower on the Salinas dataset, respectively. This result shows that it is difficult to fully extract features only relying on 2DCNN. DBDA is a model based on 3DCNN. Although it uses spatial attention mechanism and spectral attention mechanism to extract spatial and spectral features, its OA on the PU and SA datasets is 0.17% and 0.43% lower than our proposed model, respectively. The reason is that this model cannot use the global information of neighborhood pixel blocks for classification. Although, in the KSC dataset, the OA of DBDA is 0.01% higher than our proposed model, the accuracy of our proposed model on class 5 (Oak/Broadleaf) reaches 100%, while the accuracy of DBDA on class 5 is only 99.52%. The performance of our proposed model on the three datasets shows that, compared to the CNN-based model, the model that combines transformer and CNN can also reach a competitive level of accuracy.

The article "Spectral-Spatial Attention Transformer with Dense Connection for Hyperspectral Image Classification" was published in 2022. Journal: Comput Intell Neurosci.

Figures 13–15 visualize the classification results of our proposed model and the other five models on three datasets. It can be clearly seen in the classification map that there are a lot of noise points on the 1D-CNN classification map because the model does not extract the spatial features of HSI. The rest of the model used for comparison and the model we proposed all use the spatial information of HSI to help classification. Thus, the noise points problem is solved. Moreover, since M3D-DCNN, SC-FR, and pResNet do not use an attention mechanism, these models are more likely to be disturbed by pixels and spectral bands that do not contribute to the classification. For example, on the SA dataset, none of these models can accurately mark class 15 (Vinyard_untrained), and our proposed model marks class 15 most accurately. Although DBDA also uses the attention mechanism, it can be observed in the classification map that the classification effect is not as good as the model we proposed. Specifically, by comparing ground-truth images, our proposed model achieves a more accurate and smooth classification effect.

The above experiments can prove that our proposed model can achieve competitive performance compared with the CNN-based model. But balancing performance and efficiency is also important for the model.  Table 9 shows the training time and test time of pResNet, DBDA, and our proposed model on PU, KSC, and SA. Our proposed model has a decrease in training time compared with DBDA and pResNet. Although DBDA performs better on KSC than our proposed model, the training time of our proposed model is only 65% of DBDA, which shows that our model achieves a better balance between efficiency and accuracy.

### 4.2. Computing Time for Selecting Different Numbers of Bands

When we introduced the spectral-spatial attention module in Section 2, we mentioned that this module will select appropriate bands in the last layer (i.e., the 1 × 1 convolution layer) to reduce redundant information, which can also reduce the time required for the model to train and test.  Table 10 shows the training time and test time of the model when the spectral-spatial attention module selects 16, 32, and 64 bands. We can find that as the number of selected bands decreases, both the training time and the testing time of the model decrease.

The article "Spectral-Spatial Attention Transformer with Dense Connection for Hyperspectral Image Classification" was published in 2022. Journal: Comput Intell Neurosci.

### 4.3. Effectiveness of the Dense Connection

Dense connection can improve the flow of information between transformer encoder blocks and reduce the loss of information. To prove the effectiveness of dense connection, we removed dense connection and compared the performance of these two models.

Figure 16 shows the improvement of model performance by dense connections. A model with a dense connection can achieve higher accuracy. We conclude that dense connection can improve the performance of model classification.

### 4.4. Effectiveness of the Spectral-Spatial Attention Module

In Section 2, we explain the role of the CNN-based spectral-spatial attention module. To prove the effectiveness of the spectral-spatial attention module, we removed the spectral-spatial attention module, spectral attention, and spatial attention, respectively, and compared the performance of these four models.

The impact of the spectral-spatial attention module on the model performance is shown in Figure 17. The performance of the model is greatly improved by extracting low-level local features from neighborhood pixel blocks. This shows that combining the local features extracted by CNN and the global features extracted by transformer can more effectively improve the performance of the model. It is worth noting that, on the SA dataset, the accuracy of our proposed model is improved after removing the spectral attention. The reason is that many pixels with different labels in the SA dataset have similar spectral characteristics. After adding spectral attention, the model pays too much attention to the spectral features. We conclude that spectral-spatial attention module can improve the performance of model classification.

## 5. Conclusion

In this paper, we propose a model that combines transformer and a CNN-based spectral-spatial attention mechanism. This model can separately extract the local and global features of HSI. The experimental results show that the model combining transformer and CNN has better performance than the CNN-based model. The model first uses a spectral-spatial attention mechanism to extract local features and reduce the impact of redundant information on classification, then converts neighborhood pixel blocks into sequences, and extracts global features through the transformer part of the model. Finally, it is classified through the fully connected layer.

In the experiment, we first analyzed the influence of batch size, spatial size, training samples, and number of heads of the multihead self-attention mechanism on classification accuracy. Next, we compared the experimental results of our proposed model with the other five models on three public datasets. The experimental results show that, compared to several other models based entirely on CNN, the model combined with CNN and transformer also achieved competitive accuracy. Meanwhile, the experiments show that it is completely feasible to use transformer for HSI classification.

The article "Spectral-Spatial Attention Transformer with Dense Connection for Hyperspectral Image Classification" was published in 2022. Journal: Comput Intell Neurosci.

Future research should focus more on efficient transformer encoder block and attention mechanisms to process HSI information. By combining the local and global features of HSI more effectively, the accuracy of the HSI classification model can be further improved, and a more effective HSI classifier can be constructed.

## Figures and Tables

**Figure 1:** Spectral-spatial attention module.

**Figure 2:** Spectral attention module.

**Figure 3:** Spatial attention module.

**Figure 4:** The process of processing the input image into a sequence.

**Figure 5:** The structure of the transformer encoder block.

**Figure 6:** Framework of the proposed model.

**Figure 7:** Kennedy Space Center maps: (a) false-color image; (b) ground-true map.

**Figure 8:** University of Pavia maps: (a) false-color image; (b) ground-true map.

**Figure 9:** Salinas maps: (a) false-color image; (b) ground-true map.

**Figure 10:** Overall classification accuracy of different batch size.

**Figure 11:** Overall classification accuracy of different spatial sizes.

**Figure 12:** Overall classification accuracy of different number of heads.

**Figure 13:** Classification maps of the different models for the Kennedy Space Center dataset: (a) 1D-CNN, (b) M3D-DCNN, (c) SC-FR, (d) pResNet, (e) DBDA, and (f) proposed.

**Figure 14:** Classification maps of the different models for the University of Pavia dataset: (a) 1D-CNN, (b) M3D-DCNN, (c) SC-FR, (d) pResNet, (e) DBDA, and (f) proposed.

**Figure 15:** Classification maps of the different models for the Salinas dataset: (a) 1D-CNN, (b) M3D-DCNN, (c) SC-FR, (d) pResNet, (e) DBDA, and (f) proposed.

**Figure 16:** Effectiveness of the dense connections.

**Figure 17:** Effectiveness of the spectral-spatial attention module.

**Table 1:** Detailed information on three hyperspectral datasets.

	KSC	PU	SA
Type of sensor	AVIRIS	ROSIS	AVIRIS
Spatial size	512 × 614	610 × 340	512 × 217
Spectral range	0.4–2.5 *μ*m	0.43–0.86 *μ*m	0.4–2.5 *μ*m
Spatial resolution	18 m	1.3 m	3.7 m
Bands	176	103	204
Number of classes	13	9	16

**Table 2:** Samples information for the Kennedy Space Center dataset.

No.	Class	Total	Train	Test
1	Scrub	761	200	561
2	Willow swamp	243	200	43
3	CP hammock	256	200	56
4	Slash pine	252	200	52
5	Oak/broadleaf	161	129	32
6	Hardwood	229	200	29
7	Swamp	105	84	21
8	Graminoid marsh	431	200	231
9	Spartina marsh	520	200	320
10	Cattail marsh	404	200	204
11	Salt marsh	419	200	219
12	Mud flats	503	200	303
13	Water	927	200	727
Total		5211	2413	2798

The article "Spectral-Spatial Attention Transformer with Dense Connection for Hyperspectral Image Classification" was published in 2022. Journal: Comput Intell Neurosci.

**Table 3:** Samples information for the University of Pavia dataset.

No.	Class	Total	Train	Test
1	Asphalt	6631	400	6231
2	Meadows	18,649	400	18,249
3	Gravel	2099	400	1699
4	Trees	3064	400	2600
5	Sheets	1345	400	945
6	Bare soils	5029	400	4629
7	Bitumen	1330	400	930
8	Bricks	3682	400	3282
9	Shadows	947	400	547
Total		42,776	3600	39,176

**Table 4:** Samples information for the Salinas dataset.

No.	Class	Total	Train	Test
1	Brocoli_green_weeds_1	2009	201	1808
2	Brocoli_green_weeds_2	3726	373	3353
3	Fallow	1976	198	1778
4	Fallow_rough_plow	1394	140	1254
5	Fallow_smooth	2678	268	2410
6	Stubble	3959	396	3563
7	Celery	3579	358	3221
8	Grapes_untrained	11,271	1128	10143
9	Soil_vinyard_develop	6203	621	5582
10	Corn_senesced_green_weeds	3278	328	2950
11	Lettuce_romaine_4wk	1068	107	961
12	Lettuce_romaine_5wk	1927	193	1734
13	Lettuce_romaine_6wk	916	92	824
14	Lettuce_romaine_7wk	1070	107	963
15	Vinyard_untrained	7268	727	6541
16	Vinyard_vertical_trellis	1807	181	1626
Total		54,129	5418	48,711

**Table 5:** Effect evaluation of models with different training sample.

Dataset	Training sample	OA	AA	KAPPA × 100
KSC	200	99.96	99.94	99.92
KSC	300	99.94	99.80	99.93
KSC	400	99.96	99.89	99.95
PU	200	98.20	98.59	97.58
PU	300	99.39	99.59	99.17
PU	400	99.69	99.82	99.58
SA	5%	98.78	99.35	98.64
SA	10%	99.67	99.82	99.63
SA	15%	99.88	99.92	99.87

**Table 6:** Classification results of different methods for the University of Pavia dataset.

Class	1D-CNN	M3D-DCNN	SC-FR	pResNet	DBDA	Proposed
1	74.36	95.32	99.79	99.51	99.80	99.60
2	71.64	97.20	99.58	99.69	99.73	99.58
3	82.51	94.84	99.62	99.82	99.69	99.72
4	95.01	98.47	97.14	99.16	96.54	99.74
5	99.71	99.95	99.44	99.99	99.50	100.00
6	83.08	98.51	99.52	99.98	99.97	99.95
7	93.72	97.69	100.00	99.98	99.94	100.00
8	80.81	95.85	99.06	99.79	99.41	99.85
9	99.82	99.71	99.14	99.89	99.20	99.96
OA (%)	77.85 ± 1.50	97.04 ± 1.33	99.40 ± 0.28	99.69 ± 0.11	99.52 ± 0.17	**99.69** ± 0.15
Variance (OA)	2.2536	1.7582	0.0793	0.0132	0.0281	0.0226
AA (%)	86.74 ± 0.37	97.50 ± 0.87	99.26 ± 0.19	99.76 ± 0.07	99.31 ± 0.21	**99.82** ± 0.06
Variance (AA)	0.1337	0.7536	0.0372	0.0053	0.0452	0.0037
KAPPA × 100	71.40 ± 1.73	95.97 ± 1.79	99.18 ± 0.39	99.58 ± 0.16	99.34 ± 0.23	**99.58** ± 0.21

**Table 7:** Classification results of different methods for the Kennedy Space Center dataset.

Class	1D-CNN	M3D-DCNN	SC-FR	pResNet	DBDA	Proposed
1	87.81	98.75	99.45	99.84	99.91	99.84
2	84.65	98.60	100.00	100.00	100.00	100.00
3	90.71	98.39	99.82	100.00	100.00	100.00
4	57.69	93.85	100.00	98.65	99.81	99.81
5	49.69	95.62	100.00	100.00	99.69	100.00
6	60.00	98.97	100.00	100.00	100.00	100.00
7	81.90	100.00	100.00	100.00	100.00	99.52
8	88.18	99.18	99.96	100.00	100.00	100.00
9	94.12	99.84	99.88	100.00	100.00	100.00
10	95.00	99.46	100.00	100.00	100.00	100.00
11	94.79	99.91	99.95	100.00	100.00	100.00
12	88.32	99.70	100.00	100.00	100.00	100.00
13	100.00	100.00	90.00	99.92	100.00	100.00
OA (%)	91.54 ± 0.64	99.36 ± 0.25	97.27 ± 7.75	99.92 ± 0.08	**99.97** ± 0.05	99.96 ± 0.06
Variance (OA)	0.4113	0.0631	60.1004	0.0061	0.0021	0.0032
AA (%)	82.53 ± 1.63	98.64 ± 0.67	99.16 ± 2.29	99.88 ± 0.17	**99.95** ± 0.09	99.94 ± 0.12
Variance (AA)	2.6728	0.4429	5.2215	0.0288	0.0073	0.0133
KAPPA × 100	90.07 ± 0.75	99.24 ± 0.30	96.87 ± 8.87	99.91 ± 0.09	**99.97** ± 0.05	99.95 ± 0.07

The article "Spectral-Spatial Attention Transformer with Dense Connection for Hyperspectral Image Classification" was published in 2022. Journal: Comput Intell Neurosci.

**Table 8:** Classification results of different methods for the Salinas dataset.

Class	1D-CNN	M3D-DCNN	SC-FR	pResNet	DBDA	Proposed
1	84.89	99.85	99.75	100.00	100.00	100.00
2	98.17	99.97	99.80	100.00	100.00	100.00
3	89.97	99.85	99.13	99.93	100.00	100.00
4	99.51	99.63	89.39	99.97	99.69	99.74
5	97.06	97.42	99.39	99.83	97.46	99.72
6	99.76	99.99	100.00	100.00	100.00	100.00
7	99.42	99.62	100.00	99.95	100.00	99.99
8	84.76	93.23	97.23	99.21	99.39	99.21
9	98.00	99.85	99.95	99.99	100.00	100.00
10	87.53	98.17	99.43	99.51	99.69	99.84
11	74.88	98.80	98.92	99.75	99.97	99.82
12	99.50	100.00	99.99	99.99	100.00	99.98
13	97.88	99.85	99.93	99.94	100.00	99.99
14	91.10	98.81	99.73	99.98	99.83	99.80
15	56.75	88.67	96.44	98.88	96.48	99.09
16	88.18	98.60	99.69	99.90	99.99	99.91
OA (%)	87.65 ± 0.48	96.67 ± 0.58	98.51 ± 0.71	99.63 ± 0.24	99.24 ± 0.75	**99.67** ± 0.08
Variance (OA)	0.2272	0.3416	0.5099	0.0554	0.5635	0.0057
AA (%)	90.46 ± 0.65	98.27 ± 0.29	98.67 ± 1.79	99.80 ± 0.13	99.53 ± 0.34	**99.82** ± 0.05
Variance (AA)	0.4164	0.0817	3.1987	0.0171	0.1147	0.0029
KAPPA × 100	86.21 ± 0.53	96.29 ± 0.65	98.34 ± 0.80	99.59 ± 0.26	99.16 ± 0.84	**99.63** ± 0.08

**Table 9:** Training time and test time for different models on the three datasets.

		pResNet	DBDA	Proposed
University of Pavia	Training time (s)	1914.14	2416.56	**713.60**
	Test time (s)	40.68	53.30	**35.55**

Kennedy Space Center	Training time (s)	1499.25	1464.75	**959.10**
	Test time (s)	**3.76**	4.35	3.98

Salinas	Training time (s)	1972.93	1806.80	**1290.13**
	Test time (s)	**27.11**	39.62	30.520

**Table 10:** Training time and test time for selecting different numbers of bands.

Number of selected bands		KSC	PU	SA
16	Training time (s)	884.59	684.13	1128.92
	Test time (s)	3.76	33.88	29.97

32	Training time (s)	894.42	703.32	1149.99
	Test time (s)	3.79	35.72	28.29

64	Training time (s)	959.10	713.60	1290.13
	Test time (s)	3.98	35.55	30.52

## Data Availability

The data that support the findings of this study are openly available in Hyperspectral Remote Sensing Scenes at https://www.ehu.eus/ccwintco/index.php/Hyperspectral_Remote_Sensing_Scenes.
